The article "Development of Refractive Parameters in 3- to 6-Year-Old Children and Its Application in Myopia Prediction and Intervention Guidance" was retracted in 2023. Reasons: signs of a paper mill; suspected computer-generated content; unreliable results or conclusions; concerns about the data.

# Development of Refractive Parameters in 3- to 6-Year-Old Children and Its Application in Myopia Prediction and Intervention Guidance

**DOI:** 10.1155/2021/3656831

**Published:** 2021-12-16

**Authors:** Ya Zhang, Ming Su, Hua Liu, Yanxia Song, Jing Liu, Huihui Sun, Xueya Wu, Xiaoge Yang, Liqin Qi, Feifan Du, Lili Liu, Lu Chen, Jing Huang, Xiting Guo, Zhongnan Yang, Xueping Yang

**Affiliations:** ^1^The First Affiliated Hospital of Jinan University, Guangzhou 510632, China; ^2^Shijiazhuang Aier Eye Hospital, Shijiazhuang 050000, China; ^3^Hebei Children's Hospital, Shijiazhuang 050000, China; ^4^Jinan University, Guangzhou 510632, China; ^5^The Third Affiliated Hospital of Jinzhou Medical University, Jinzhou 121000, China; ^6^Hebei Women and Children Health Care Center, 050000, China; ^7^Baoding Aier Eye Hospital, 071000, China; ^8^Cangzhou Aier Eye Hospital, 061000, China; ^9^Qinhuangdao Aier Eye Hospital, Qinhuangdao 066000, China

## Abstract

**Objective:**

To investigate refractive development and prevalence of myopia in children aged 3-6 years in Hebei Province, China, and to explore the developmental law of refraction, so as to clinically guide the prediction and intervention of myopia.

**Methods:**

In May 2019, a total of 6120 people were inspected in 68 kindergartens in 11 cities in Hebei Province. Child refractive refraction was checked under noncycloplegia using a handheld binocular vision screener (SW-800, SUOER, Tianjin, China). Axial length (AL) and corneal radius of curvature (CR) were measured using an ocular biometry (IOLMaster 500, Carl Zeiss, Germany). Myopia was defined as spherical equivalent (SE) ≤ −0.75 D.

**Results:**

A total of 5506 children aged 3-6 years met the criteria and were included in the statistical analysis. The prevalence of myopia was 3.49% (1.93% at age 3, 2.90% at age 4, 3.78% at age 5, and 3.88% at age 6). Overall, the mean SE was +0.67 ± 1.05 D (+0.81 ± 1.00 D at age 3, +0.79 ± 1.05 D at age 4, +0.67 ± 1.08 D at age 5, and +0.13 ± 1.01 D at age 6); the mean CR was 7.76 ± 0.26 mm (7.78 ± 0.26 mm at age3, 7.75 ± 0.25 mm at age 4, 7.77 ± 0.26 mm at age 5, and 7.76 ± 0.25 mm at age 6); the mean AL was 22.31 ± 0.73 mm (21.98 ± 0.63 mm at age 3, 22.12 ± 0.69 mm at age 4, 22.34 ± 0.73 mm at age 5, and 22.49 ± 0.73 mm at age 6).

**Conclusions:**

Prevalence of myopia increases with age in children aged 3-6 years in Hebei, China. With the increase of age, CR is basically stable, and AL increases gradually. AL/CR, which is closely related to SE, can be used as an indicator to predict myopia and guide clinical work.

## 1. Introduction

The refractive state of the newborn is mostly hyperopia. The transition from hyperopia to emmetropia with age is called emmetropization. Preschool age is a critical period of children's eye development; refractive development state during this period will fundamentally affect the process of emmetropization. Early emmetropization can lead to the development of refractive state to myopia. Myopia is a public health problem in China and other countries in East Asia [1]. In recent years, myopia presents two trends, that is, the prevalence increases year by year and the age of onset of myopia decreases gradually. Earlier onset age increases the difficulty to control degrees of myopia and the probability of developing into high myopia. Patients with high myopia carry higher risk of complications such as macular disease, retinal detachment, and choroidal neovascularization and are associated with worse prognosis. Therefore, it is necessary to start to focus on the refractive development of children at the preschool age. Studies on the prevalence of ametropia in preschool children have been published successively in Chinese cities such as Hong Kong [2] (2004), Guangzhou [3] (2013), Xuzhou [4] (2014), Shenzhen [5] (2017), and Shanghai [6] (2018). However, there are still no reports on refractive data of preschoolers covering the whole province. Hebei Province is one of the main provinces in North China. This baseline survey was conducted on the refractive status and ocular biological characteristics of preschool children in 11 cities in Hebei Province. We aim to provide basic data for the prevention and control of myopia in the whole province and even the country.

Accommodation is high in children, and therefore, cycloplegic refraction is considered as the gold standard to evaluate children's refractive error [7, 8]. However, cycloplegic refraction is less accepted by children and their guardians because ciliary muscle paralysis may bring near vision unclear, photophobia, allergy, and other reactions within a certain period of time, affecting normal life [9]. Thus, the proportion of cycloplegic refraction in preschool children decreases. To avoid decreasing participation rate, researchers usually avoid ciliary muscle paralysis and select the applicable automatic optometric devices for measurements when allowed [10].

Currently, handheld binocular vision screener is widely used for refractive screening of preschool children internationally [11–13]. This device screens both eyes at once from a 1–3 meter distance using the built-in fogging technique. Compared with the desktop computer optometry instrument, this handheld one can eliminate the near perception adjustment. Moreover, this is an efficient and safe noninvasive method widely used in refractive screening in preschoolers [14, 15]. In addition to the measurement tools used, the prevalence of refractive error is also affected by the threshold setting [16]. The International Myopia Institute (IMI) has suggested that the threshold for myopia in the absence of cycloplegia (spherical equivalent (SE) ≤ −0.75 D or SE ≤ −1.00 D) is higher than the consensus threshold value for myopia under cycloplegia (SE ≤ −0.50 D) [17].

When cycloplegic refraction is difficult to perform, axial length (AL)/corneal radius of curvature (CR) may be the second choice to predict SE, estimating child refractive values based on the ratio of AL to CR [18]. Ocular biometry can provide reliable ocular parameters of children. AL is positively correlated with retinal complications of high myopia. Despite the importance of the eye axis, few eye axis-based population studies exist for preschool children [19–22]. This study involves pediatric ocular biometry measurements such as AL and CR. Based on the collected data, we aimed to comprehensively understand the refractive development of preschool children aged 3-6 years in Hebei Province and then clinically guide the myopia prediction and intervention of preschoolers.

## 2. Materials and Methods

### 2.1. Study Population

Hebei Province is located in the North China Plain with an area of 188,800 square kilometers, embracing the capital Beijing, adjacent to Tianjin to the east and close to Bohai Sea. It is an important administrative area for the coordinated development of the Beijing-Tianjin-Hebei region. In 2020, Hebei had a permanent resident population of 74,610,200. Hebei has 11 cities including the provincial capital Shijiazhuang, Tangshan, Qinhuangdao, Handan, Xingtai, Baoding, Zhangjiakou, Chengde, Cangzhou, Langfang, and Hengshui. This study, based on the results of baseline survey on refractive development of preschoolers in Hebei Province, covered all 11 cities and was jointly completed by Aier Eye Hospital in Hebei Province, Children's Hospital of Hebei Province, and municipal maternal and child healthcare institutions in May 2019. A total of 6120 preschoolers from 63 kindergartens were investigated. The inclusion criteria were as follows: (1) all inspections shall be conducted; (2) same inspection items, at least three measurement results, and good repeatability of data; (3) no obvious strabismus or other ocular organic lesions. The exclusion criteria of the subjects were as follows: (1) children with a missing inspection item, (2) children whose data was recorded incorrectly, and (3) children who used any eye drops or oral medicine within 1 month prior to the examination.

### 2.2. Examination

One pediatric ophthalmologist, two ophthalmic assistants, and one outreach worker were selected from Aier Eye Hospital in each city involved in the survey. A total of 55 people from 11 cities were trained intensively. There were unified standards for operation procedures, diagnosis, and record format. Two ophthalmic assistants, respectively, performed refractive screening and obtained ocular biometric measurements. One ophthalmologist examined eye position, eye movement, anterior segment, and eye fundus. Refractive screening was carried out in a dark area with an examination distance of about 1 meter. A binocular vision screener (SW-800, SUOER, Tianjin, China) was used in every city, calibrated by the same engineer one week before the start of the initial investigation. The device was checked by ophthalmic assistants before each survey to ensure the relative accuracy of the screener. The results of at least three measurements must be consistent to be adopted. This meant that the difference of spherical or cylindrical power in each measurement must be <0.50 D or will be remeasured. Children avoided short-distance use of eyes within half an hour before the refractive examination. AL and CR were measured in a noncontact manner (IOLMaster 500, Carl Zeiss Meditec, Oberkochen, Germany). The average of five consecutive measurements was calculated, and the images with the highest signal-to-noise ratio were chosen to ensure a robust assessment of AL. In order to avoid affecting the accuracy of the visual examination due to the instrument light source, the eye position, eye movement, anterior segment, and eye fundus were finally examined by the pediatric ophthalmologist. The anterior segment was examined using a desktop slit-lamp microscope (SL-D4 Topcon Japan), while the eye fundus using direct ophthalmoscope (vision YZ 6f, Suzhou 66, China).

### 2.3. Recording Methods and Definition

The calculation formula of SE was SE = sphere + 1/2 cylinder. According to the SE value, the included preschoolers were divided into four groups: myopia (SE ≤ −0.75 D), emmetropia (−0.75 D < SE < +0.50 D), mild hyperopia (+0.50 D ≤ SE < +2.00 D), and hyperopia (SE ≥ +2.00 D). The calculation formula of CR was CR = (CR_1_ + CR_2_)/2, where CR_1_ = 337; 5/flat corneal curvature; CR_2_ = 337; 5/steep corneal curvature. AL/CR represented the ratio of AL to CR.

### 2.4. Statistical Method

Statistical analysis was performed using the IBM SPSS 23. 0. For comparison of each parameter in different genders and ages, the independent sample *U* test was used for data satisfying the Gaussian distribution with homogeneity of variance, while the Wilcoxon rank sum test for data not satisfying the Gaussian distribution and Dunn-Bonferroni correction for comparison of each two groups.

Differences in prevalence of refractive error between boys and girls were determined by Pearson chi-square test. Scatter plots and Pearson correlation were used to analyze linear relationship between AL and CR, age, and sex, respectively. Subsequently, regression analysis was carried out. All *P* values were two-sided with test level *α* = 0.05 and *P* < 0.05 considered statistically significant.

## 3. Results

### 3.1. Study Population

A total of 6120 people were inspected from 68 kindergartens in 11 cities (regions) in Hebei Province. After exclusion of the invalid data, a total of 5506 people were included in the statistics. The demographic characteristics of the subjects are shown in Table 1. The average age was 4.94 ± 0.87 years, and the average monthly age was 64.10 ± 9.99 months (ranging from 36 to 83 months).

### 3.2. Measurement Agreement

Correlation analysis was conducted on the right eye data and the left eye data, respectively, and high consistency between the two eyes was obtained (correlation coefficient SE: *r* = 0.754, *P* ≤ 0.001; AL: *r* = 0.952, *P* ≤ 0.001; CR: *r* = 0.960, *P* ≤ 0.001). Right eye data were randomly selected for statistics.

### 3.3. Diopter

The average of overall SE was +0.67±1.05 D (median: +0.25 D; interquartile range: -0.13 to +1.63 D) (Table 2). Overall and different gender children aged 3-6 showed a decreasing trend with age (Figure 1). Additionally, the differences of SE values were statistically significant among different age groups (in total population: overall *P* < 0.001, *P* = 0.879 for 3- vs. 4-year-old group, *P* = 0.001 for 3- and 5-year-old group, *P* = 0.002 for 3- vs. 6-year-old group, *P* = 0.001 for 4- vs. 5-year-old group, *P* < 0.001 for 4- vs. 6-year-old group, *P* = 0.006 for 5- vs. 6-year-old group; in boys, overall *P* < 0.001, *P* = 0.775 for 3- vs. 4-year-old group, *P* < 0.001 for 3- vs. 5-year-old group, *P* = 0.026 for 3- vs. 6-year-old, *P* < 0.001 for 4- vs. 5-year-old group, *P* < 0.001 for 4- vs. 6-year-old, *P* = 0.362 for 5- vs. 6-year-old group; in girls, overall *P* = 0.001, *P* = 0.916 for 3- vs. 4-year-old group, *P* = 0.671 for 3- vs. 5-year-old group, *P* = 0.031 for 3- vs. 6-year-old group, *P* = 0.468 for 4- vs. 5-year-old group, *P* < 0.001 for 4- vs. 6-year-old group, *P* = 0.002 for 5- vs. 6-year-old group). Among children aged 3-6 years, the SE value of girls was higher than that of boys, and the difference was statistically significant (overall: *P* = 0.013 < 0.05, 3-year-old group: *P* = 0.841, 4-year-old group: *P* = 0.866, 5-year-old group: *P* = 0.001, and 6-year-old group: *P* = 0.337).

### 3.4. Ocular Biometric Measurements

Biometric parameters of the eyes were measured in different ages and different genders (Table 3), and the results showed that AL was in normal distribution, while CR and AL/CR were approximately in normal distribution (Figures 2(a)–2(c)).

In the total population, the average of AL was 22.31 ± 0.73 mm, and AL increased gradually with age (Figure 3(a)); the differences between different age groups were statistically significant (overall *P* < 0.001, *P* = 0.001 for age 3 vs. age 4, *P* < 0.001 for age 3 vs. age 5, *P* < 0.001 for age 3 vs. age 6, *P* < 0.001 for age 4 vs. age 5, *P* < 0.001 for age 4 vs. age 6, and *P* < 0.001 for age 5 vs. age 6). The average AL of girls (22.03 ± 0.68 mm) was significantly lower than that of boys (22.57 ± 0.68 mm); the difference was statistically significant between girls and boys (overall: *P* < 0.001, 3-year-old group: *P* < 0.001, 4-year-old group: *P* < 0.001, 5-year-old group: *P* < 0.001, and 6-year-old group: *P* < 0.001).

The average CR was 7.76 ± 0.26 mm, and CR showed no significant change with age (*P* = 0.106) (Figure 3(b)). The average CR value of boys (7.83 ± 0.25 mm) was higher than that of girls (7.70 ± 0.25 mm), and the difference between male and female was statistically significant (overall: *P* < 0.001, 3-year-old group: *P* < 0.001, 4-year-old group: *P* < 0.001, 5-year-old group: *P* < 0.001, and 6-year-old group: *P* < 0.001).

The average AL/CR was 2.87 ± 0.08. With the increase of age, AL/CR gradually increased (Figure 3(c)), and the differences between different age groups were statistically significant (overall *P* < 0.001, *P* < 0.001 for age 3 vs. age 4, *P* < 0.001 for age 3 vs. age 5, *P* < 0.001 for age 3 vs. age 6, *P* < 0.001 for age 4 vs. age 5, *P* < 0.001 for age 4 vs. age 6, and *P* < 0.001 for age 5 vs. age 6). The average AL/CR of boys (2.88 ± 0.08 mm) was higher than that of girls (2.86 ± 0.07 mm), and the difference was statistically significant (overall *P* < 0.001, *P* = 0.317 in the 3-year-old group, *P* < 0.001 in the 4-year-old group, *P* < 0.001 in the 5-year-old group, and *P* < 0.001 in the 6-year-old group).

### 3.5. Correlation Regression Analysis

AL was positively correlated with age (*r* = 0.218, *P* ≤ 0.001), CR (*r* = 0.694, *P* ≤ 0.001), and sex (boy = 1, girl = 0; *r* = 0.373, *P* ≤ 0.001), respectively (Figures 4(a)–4(c)). Further, multiple linear regression models showed the relationship between AL and age, CR, and sex (boy = 1, girl = 0): *R*^2^ = 0.551, AL = 0.3∗Sex + 0.177∗Age + 1.798∗CR + 7.321 (*P* ≤ 0.001) (Table 4) (Figure 4(d)). This meant that male, older age, and higher CR value were all factors leading to longer AL.

### 3.6. Diopter and Ocular Biometric Measurements

Among different refractive types, the larger AL/CR is, the lower the positive spherical mirror of SE is (Figures 5(a) and 5(b)). In the overall emmetropia group, the mean of AL/CR was 2.88 (2.89 for boys and 2.87 for girls) and the mean of SE was -0.06 D (-0.06 D for boys and -0.05 D for girls). In the overall myopia group, AL/CR average was 2.93 (2.94 for boys and 2.92 for girls), and SE average was -1.25 D (-1.30 D for boys and -1.17 D for girls) (Table 5).

### 3.7. Prevalence of Refractive Error

The prevalence of myopia in children was 3.49% (1.93% in the 3-year-old group, 2.90% in the 4-year-old group, 3.78% in the 5-year-old group, and 3.88% in the 6-year-old group) (Table 6). The prevalence of myopia increased with age, in preschoolers, and there was statistically significant difference among different age groups (*P* ≤ 0.001). Additionally, compared with girls, boys had a significantly higher prevalence of myopia, but a lower prevalence of hyperopia (both *P* ≤ 0.001, Table 6). In the total number of children, emmetropia accounted for the largest proportion (51.36%), followed by mild hyperopia (36.67%) (Figure 6), indicating that more than half of preschool children entered emmetropia.

## 4. Discussion

This baseline survey revealed that in the absence of cycloplegia, the average SE of 3- to 6-year-old children in Hebei Province of China was 0.67 ± 1.05 D (median: +0.25D). This SE value was lower than that previously reported in 3- to 6-year-old children receiving 1% cyclopentolate in Shanghai (+1.20 ± 1.05 D) [6], Shenzhen (1.37 ± 0.63 D) [5], and Guangzhou (+1.42 ± 0.79 D) [3]. In 2019, Li et al. [23] reported that the median SE of children aged 4-6 in Shanghai under nonmydriatic condition was +0.25 D, which was consistent with this study. The results of Shandong children's ophthalmology study in 2015 showed that the difference of SE value between cycloplegia and noncycloplegia in children aged 4-18 was 0.78 ± 0.79 D [10], which was consistent with the SE difference between this study (noncycloplegia) and the previous reports (cycloplegia). In this study, SE values of 4- to 6-year-old children gradually decreased with age, and the difference was statistically significant, but the diopter changed very little with age [3]. SE of the 3-year-old group was little higher than that of the 4-year-old group with no significant difference, which is considered that in the noncycloplegic state, children aged 3 years may be more affected by accommodation. A binocular vision screener, with accuracy, rapidity, maneuverability, and repeatability for detecting diopter under nonmydriatic state, has gradually been recognized by more and more researchers. Moreover, this device has obtained approval of the Food and Drug Administration (FDA) [24]. However, this kind of screener does reduce its accuracy due to the effect of strong accommodation in younger children, and then, the prevalence of myopia will be overestimated in younger children [10, 25–28]. The Sankara Nethralaya Tamil Nadu Essilor Myopia (STEM) study [16] pointed out that in noncycloplegic refraction using an open-field autorefractor, the threshold of SE ≤ −0.75 D was equivalent to the threshold value for myopia under cycloplegia (SE ≤ −0.50 D). Therefore, changing the threshold for myopia can reduce the influence of accommodation on the prevalence of myopia under cycloplegia to some extent. In this study, when myopia was defined as SE ≤ −0.75 D, the overall prevalence of myopia in children aged 3-6 years was 3.49% and 3.88% in children aged 6 years. Similarly, in 2017, Guo et al. [5] obtained the prevalence rate of myopia (3.7%) among children aged 3-6 years after cycloplegia (1% cyclopentolate) in 8 kindergartens in Shenzhen. Additionally, the mean SE of boys (0.64 ± 1.04 D) was lower than that of girls (0.72 ± 1.06 D), and the difference was statistically significant (*P* = 0.013 < 0.05). The prevalence of myopia in boys (4.00%) was higher than that in girls (3.06%), but there was no significant difference between genders (*P* = 0.061 > 0.05). In preschool period, the main refractive state is emmetropia (51.67%) in children, but boys should be paid more attention than girls in the prevention and control of myopia.

In this study, the average AL value of preschoolers aged 3-6 years in Hebei Province was 22.31 ± 0.73 mm, and the average CR was 7.76 ± 0.26 mm, which is highly consistent with the data of Shenzhen (AL: 22.39 ± 0.68 mm, CR; 7.79 ± 0.25 mm) [5] and the data of Shanghai (AL: 22.36 ± 0.72 mm, CR: 7.83 ± 0.25 mm) [20]. We also found that AL has a linear relationship with age, CR, and gender, respectively. And multiple linear regression model further revealed that older age or higher CR value was associated with longer AL; AL of boys was about 0.3 mm longer than that of girls at the same age (*R*^2^ = 0.551, AL = 0.3∗gender + 0.177∗age + 1.798∗CR + 7.321). It has been reported that in children aged 6-12, male AL is 0.5 mm longer than female AL [26]. It suggests that the AL difference between males and females gradually increases with age, which further indicates that males have a larger increase of AL than females [27]. The longer the AL, the higher the chance of fundus lesions [29]. This survey results suggest that, if AL cannot be examined due to objective factors, we can speculate AL according to the CR value, gender, and age obtained by an autorefractor and therefore can provide preliminary myopia prediction and intervention.

The correlation between AL/CR and ametropia was first proposed by Grosvenor and Scott [30]. Small changes in AL/CR will lead to significant changes in ametropia, and the correlation between ametropia and AL/CR is significantly stronger than that between ametropia and AL or CR alone [31]. In this study, the mean SE of the emmetropia group was -0.06±0.25 D (approximately flat diopter), and the corresponding AL/CR was 2.88. When the mean SE was -0.75 D, the corresponding AL/CR was 2.89, suggesting that 2.89 can be used as a clinical myopia warning value for children aged 3-6 years. If the value is higher than this value, the possibility of myopia refractive state is very high, and the probability of high myopia can be predicted in the future. This part of the population is the most important object of myopia prevention and control. In our study, it is lower than previous reports in which the incidence of myopia is significantly increased when AL/CR > 3.0 [30, 32]. This reminds us that the adult standard cannot be used to predict myopia in preschool children. Clinically, AL/CR can be used as an index to evaluate refractive development of preschool children in the absence of cycloplegia [7]. For children aged 3-6 years with AL/CR exceeding the warning value of their corresponding age and gender, doctors make medical advice inclined to cycloplegia (excluding mydriasis contraindications) in combination with the visual acuity and autorefractor results and take comprehensive myopia prevention and control measures.

This study is the first baseline survey of preschool children, covering all 11 cities in Hebei Province. We determined the number of children receiving screening according to the population ratio, including children from public and private kindergartens in urban or county. This was to minimize the impact of region, urban or rural areas, and nature of kindergarten on the survey results, as far as possible to truly reflect the refractive development status of preschoolers in Hebei Province. Finally, this study screened a total of 6120 preschool children. The number of screenings, regional span, and reasonable population proportion are rarely in the reports of preschool children. However, there is also a limitation in this paper. Specifically, cycloplegic refraction is not used in our study in order to achieve large-scale screening and ensure the compliance of children and their parents, resulting in reduced accuracy of refractive error and the possibility of negative overcorrection error or refraction [33]. Therefore, this limitation may lead to overestimation of myopia and underestimation of hyperopia [34, 35].

In short, the age of 3-6 is a critical period of childhood eye development; the age of myopia or duration of myopia progress is the most important predictor of high myopia [36]. This large sample survey provides data related to refractive development in preschoolers aged 3-6 years. The survey is close to the situation encountered in our daily treatment, that is, we should first detect the refractive status of children in the noncycloplegic state, then explain to parents the results in combination with ocular biometric measurements, and finally decide whether mydriasis and active myopia prevention and control measures are needed. The results of this investigation are of great reference significance in future clinical work.

## 5. Conclusions

The prevalence of myopia in children aged 3-6 is increasing with age and is higher in boys than girls. Boys have longer AL and flat corneal curvature compared with girls. With the increase of age, AL and AL/CR increased gradually, and the corneal curvature was basically stable. AL/CR can be used as a predictor of myopia in children aged 3-6 years. The results of our study can play a guiding role in the prediction and intervention of myopia in children aged 3-6 years in the future clinical work.

## Figures and Tables

**Figure 1:** Average spherical equivalent (SE) for different AGE and SEX.

**Figure 2:** Distribution histograms of (a) mean axial length (AL), (b) mean corneal radius of curvature (CR), and (c) mean AL/CR.

**Figure 3:** (a) Mean axial length (AL), (b) mean corneal radius of curvature (CR), and (c) mean AL/CR trend with age.

**Figure 4:** Linear regression relationship between AL and (a) age, (b) CR, and (c) sex. (d) Multiple linear regression models showed the relationship between AL and age, CR, and sex.

**Figure 5:** (a, b) The average of SE and AL/CR in different refractive types.

**Figure 6:** Distribution of refractive types for each age group.

**Table 1:** Age and gender ratio of the participants.

Age (year)	Case (*n*)	Age (median, month)	Age (IRQ, month)	Number of boys (%)	Number of girls (%)
Total	5506	64	57-72	2828 (51.36)	2678 (48.64)
3	259	45	43-46	125 (2.27)	134 (2.43)
4	1483	54	51-57	756 (13.73)	727 (13.20)
5	2115	64	61-68	1107 (20.11)	1008 (18.31)
6	1649	75	73-78	840 (15.25)	809 (14.70)

IRQ: interquartile range.

**Table 2:** Distribution of spherical equivalent (SE) for different ages and genders.

Age (year)	Case (*n*)	Mean	Standard Deviation	Median (D)	25% (D)	75% (D)	Range (D)	Peak Degree (D)	Partial Degree (D)
Total	5506	0.67	1.05	+0.25	-0.13	+1.63	-7.50~+9.00	2.52	0.46
3	259	0.67	1.01	+0.25	-0.13	+1.63	-2.13~+5.59	0.84	0.62
4	1483	0.79	1.05	+0.50	-0.09	+1.67	-4.88~+6.59	1.29	0.27
5	2115	0.67	1.08	+0.25	-0.13	+1.63	-7.50~+9.00	3.74	0.51
6	1649	0.56	1.00	+0.13	-0.13	+1.63	-5.25~+6.88	2.17	0.55
*P* value	*P* = 0.000								
Male	2828	0.63	1.04	+0.25	-0.13	+1.63	-5.25~+6.88	3.37	-1.20
3	125	0.68	1.06	+0.25	-0.09	+1.63	-2.13~+5.59	2.30	0.93
4	756	0.80	1.08	+0.50	-0.09	+1.67	-4.88~+6.59	2.42	0.21
5	1107	0.59	1.03	+0.25	-0.13	+1.63	-3.75~+4.75	0.10	0.33
6	840	0.54	1.02	+0.13	-1.00	-0.25	-5.25~+6.88	2.94	0.41
*P* value	*P* = 0.000								
Female	2678	0.71	1.05	+0.25	-1.00	-0.25	-7.50~+9.00	3.40	0.57
3	134	0.67	0.96	+0.25	-0.13	+1.63	-1.50~+3.00	-1.18	0.23
4	727	0.78	1.00	+0.38	-0.13	+1.67	-2.63~+5.38	-0.27	0.34
5	1008	0.76	1.14	+0.38	-0.13	+1.66	-7.50~+9.00	6.26	0.61
6	809	0.59	0.99	+0.25	-0.	+1.63	-2.83~+6.13	1.27	0.72
*P* value	*P* = 0.001								
^∗^ *P* value	*P* = 0.013								

Note: *P* is the satistical difference between 3-6 years old children (Kruskal-Wallis Test). ^∗^*P* is the statistical difference between all boys and all girls aged 3-6 years (Kruskal-Wallis Test).

**Table 3:** Distribution of axial length (AL), corneal radius of curvature (CR), and AL/CR in different ages and genders.

		AL				CR				AL/CR			
Age (year)	Case (*n*)	Mean	Standard deviation	Peak degree	Partial degree	Mean	Standard deviation	Peak degree	Partial degree	Mean	Standard deviation	Peak degree	Partial degree
Total	5506	22.31	0.73	0.50	0.034	7.76	0.26	0.15	0.07	2.87	0.08	0.91	-0.04
3	259	21.98	0.63	-0.17	0.14	7.78	0.26	0.28	0.40	2.83	0.07	0.87	-0.06
4	1483	22.12	0.69	0.88	0.08	7.75	0.25	0.26	0.11	2.85	0.08	3.29	0.06
5	2115	22.34	0.73	0.67	0.01	7.77	0.26	0.15	-0.02	2.88	0.08	4.3	-0.01
6	1649	22.49	0.73	0.40	-0.07	7.76	0.25	0.04	0.09	2.90	0.07	1.66	-0.3
*P* value		*P* ≤ 0.001				*P* = 0.106				*P* ≤ 0.001			
Male	2828	22.57	0.68	0.85	0.09	7.83	0.25	0.06	0.15	2.88	0.08	2.85	0.05
3	125	22.20	0.62	-0.05	0.05	7.84	0.26	-0.10	0.30	2.83	0.07	-0.40	0.08
4	756	22.36	0.65	1.06	0.37	7.82	0.24	0.15	0.30	2.86	0.07	5.28	0.35
5	1107	22.62	0.67	1.54	0.00	7.84	0.25	0.02	0.11	2.89	0.08	4.19	0.02
6	840	22.75	0.67	0.72	-0.05	7.82	0.25	0.07	0.06	2.91	0.07	1.73	-0.24
*P* value		*P* ≤ 0.001				*P* = 0.113				*P* ≤ 0.001			
Female	2678	22.03	0.68	0.39	-0.03	7.70	0.25	0.16	0.02	2.86	0.07	2.43	-0.18
3	134	21.77	0.57	-0.28	0.12	7.72	0.26	1.03	0.57	2.82	0.07	2.08	-0.18
4	727	21.87	0.64	0.40	-0.22	7.69	0.25	0.21	0.04	2.85	0.07	1.38	-0.19
5	1008	22.04	0.67	0.43	0.02	7.70	0.25	0.07	-0.13	2.87	0.07	4.75	-0.12
6	809	22.21	0.68	0.42	-0.08	7.70	0.24	0.06	0.09	2.89	0.07	1.69	-0.40
*P* value		*P* ≤ 0.001				*P* = 0.688				*P* ≤ 0.001			
^∗^ *P* value		*P* ≤ 0.001				*P* ≤ 0.001				*P* ≤ 0.001			

Note: *P* is the statistical difference between 3- and 6-year-old children (Kruskal-Wallis test). ^∗^*P* is the statistical difference between all boys and all girls aged 3-6 years (Kruskal-Wallis test).

**Table 4:** Linear regression analysis of axial length (AL) with age, corneal radius of curvature (CR), and sex.

Coefficient^a^					
Model	Unstandardized coefficients		Standardized coefficients	*t*	Sig.
	*B*	SE	Beta		
Constant	7.321	0.209		35.074	0.000
CR	1.798	0.027	0.630	67.455	0.000
Sex	0.300	0.014	0.205	21.949	0.000
Age	0.177	0.008	0.210	23.224	0.000

^a^Dependent variable: axial length (AL); *B*: regression coefficient.

**Table 5:** The average of SE and AL/CR in different refractive types.

	Myopia				Emmetropia				Mildhyperopia				Hyperopia			
	SE		AL/CR		SE		AL/CR		SE		AL/CR		SE		AL/CR	
	Mean	Standard Deviation	Mean	Standard Deviation	Mean	Standard Deviation	Mean	Standard Deviation	Mean	Standard Deviation	Mean	Standard Deviation	Mean	Standard Deviation	Mean	Standard Deviation
Total	-1.25	0.86	2.93	0.11	-0.06	0.25	2.88	0.07	1.47	0.44	2.87	0.07	2.48	0.82	2.82	0.09
Male	-1.30	0.84	2.94	0.10	-0.06	0.25	2.89	0.07	1.48	0.44	2.88	0.07	2.47	0.77	2.83	0.09
Female	-1.17	0.89	2.92	0.11	-0.05	0.25	2.89	0.07	1.47	0.44	2.86	0.06	2.50	0.85	2.82	0.10

**Table 6:** Prevalence of refractive error.

		Myopia			Emmetropia			Mild hyperopia			Hyperopia		
Variable	Total (*n*)	Case (*n*)	Occupy (%)	95% CI	Case (*n*)	Occupy (%)	95% CI	Case (*n*)	Occupy (%)	95% CI	Case (*n*)	Occupy (%)	95% CI
Age (years)	5506	192	3.49	-1.37~-1.12	2828	51.36	-0.07~-0.05	2019	36.67	+1.46~+1.49	467	8.48	+2.41~+2.56
3	259	5	1.93	-1.06~-0.68	118	45.56	-0.14~-0.04	118	45.56	+1.45~+1.59	18	6.95	+2.08~+2.92
4	1483	43	2.90	-1.51~-0.96	689	46.46	-0.07~-0.03	607	40.93	+1.45~+1.52	144	9.71	+2.34~+2.58
5	2115	80	3.78	-1.50~-1.09	1093	51.68	-0.08~-0.05	744	35.18	+1.44~+1.51	198	9.36	+2.39~+2.63
6	1649	64	3.88	-1.41~-1.01	928	56.28	-0.07~-0.04	550	33.35	+1.41~+1.49	107	6.49	+2.31~+2.62
*P* value			*P* ≤ 0.001			*P* ≤ 0.001			*P* ≤ 0.001			*P* ≤ 0.001	
Gender													
Male	2828	111	3.93	-1.46~-1.14	1477	52.22	-0.08~-0.05	1025	36.24	+1.45~+1.51	215	7.60	+2.36~+2.57
Female	2678	81	3.02	-1.36~-0.97	1351	50.45	-0.07~-0.04	994	37.12	+1.44~+1.50	252	9.41	+2.39~+2.61
*P* value			^∗^ *P* ≤ 0.001			^∗^ *P* ≤ 0.001			^∗^ *P* ≤ 0.001			^∗^ *P* ≤ 0.001	

Note: *P* is the statistical difference between 3- and 6-year-old children (chi-square test). ^∗^*P* is the statistical difference between all boys and all girls aged 3-6 years (chi-square test).

## Data Availability

The data used to support the findings of this study are available from the corresponding author upon request.
